# Complete pathological response (ypT0N0M0) after preoperative chemotherapy alone for stage IV rectal cancer

**DOI:** 10.1186/1471-2482-14-4

**Published:** 2014-01-17

**Authors:** Surennaidoo P Naiken, Christian Toso, Laura Rubbia-Brandt, Theodoros Thomopoulos, Arnaud Roth, Gilles Mentha, Philippe Morel, Pascal Gervaz

**Affiliations:** 1 Services de chirurgie viscérale et transplantation, Département de chirurgie, Hôpitaux Universitaires de Genève, Rue Gabrielle-Perret-Gentil 4, Genève 14 1211, Suisse; 2 Services de pathologie clinique, Hôpitaux Universitaires de Genève, Rue Gabrielle-Perret-Gentil 4, Genève 14 1211, Suisse; 3 Service d’oncochirurgie, Hôpitaux Universitaires de Genève, Rue Gabrielle-Perret-Gentil 4, Genève 14 1211, Suisse

**Keywords:** Pathological complete response, Stage iv rectal cancer, Preoperative chemotherapy, Oxaliplatin

## Abstract

**Background:**

Complete pathological response occurs in 10–20% of patients with rectal cancer who are treated with neoadjuvant chemoradiation therapy prior to pelvic surgery. The possibility that complete pathological response of rectal cancer can also occur with neoadjuvant chemotherapy alone (without radiation) is an intriguing hypothesis.

**Case presentation:**

A 66-year old man presented an adenocarcinoma of the rectum with nine liver metastases (T3N1M1). He was included in a reverse treatment, aiming at first downsizing the liver metastases by chemotherapy, and subsequently performing the liver surgery prior to the rectum resection. The neoadjuvant chemotherapy consisted in a combination of oxaliplatin, 5-FU, irinotecan, leucovorin and bevacizumab (OCFL-B). After a right portal embolization, an extended right liver lobectomy was performed. On the final histopathological analysis, all lesions were fibrotic, devoid of any viable cancer cells. One month after liver surgery, the rectoscopic examination showed a near-total response of the primary rectal adenocarcinoma, which convinced the colorectal surgeon to perform the low anterior resection without preoperative radiation therapy. Macroscopically, a fibrous scar was observed at the level of the previously documented tumour, and the histological examination of the surgical specimen did not reveal any malignant cells in the rectal wall as well as in the mesorectum. All 15 resected lymph nodes were free of tumour, and the final tumour stage was ypT0N0M0. Clinical outcome was excellent, and the patient is currently alive 5 years after the first surgery without evidence of recurrence.

**Conclusion:**

The presented patient with stage IV rectal cancer and liver metastases was in a unique situation linked to its inclusion in a reversed treatment and the use of neoadjuvant chemotherapy alone. The observed achievement of a complete pathological response after chemotherapy should promote the design of prospective randomized studies to evaluate the benefits of chemotherapy alone in patients with stages II-III rectal adenocarcinoma (without metastasis).

## Background

Colorectal cancer (CRC) is a major public health problem [1,2]. Over the last two decades, its management has improved significantly, in parallel to the implementation of dedicated multidisciplinary oncological rounds [3,4]. Routine staging is now in place in almost all centers with the use of MRI and/or endo-rectal ultrasonography. Surgery has been standardized thanks to the popularization of the total mesorectal excision technique. In addition, neoadjuvant treatment has been refined with the use of chemoradiotherapy (CRT) in selected patients with locally advanced cancer. More recently, the survival of patients with metastatic rectal cancer has also improved thanks to the availability of new potent drug combinations.

To illustrate these improvements in the (neo-) adjuvant treatments, up to 10% of patients with stage IV CRC do not have detectable liver metastasis anymore on pathology following chemotherapy [5,6]. Pathologic complete response (pCR) also occurs in 10-20% of patients with rectal cancer who are treated with neoadjuvant chemo radiotherapy prior to pelvic surgery [7]. The current standard management of patients with rectal cancer reaching the peri-rectal fat (cT3-T4N0) and/or with a clinical evidence of lymphnode invasion (cTxN1) includes a neoadjuvant chemoradiotherapy [8]. At our institution, for patients with advanced synchronous colorectal liver metastasis (CRLM) and a non- obstructive primary tumor, a reversed protocol [9,10] is recommended. They include patients with multiple, often large metastases not accessible for minor (up to two segments) up-front liver resection [10]. This strategy controls the CRLM and the primary tumour, hence increasing the curative liver metastatic resection. In our initial study [11], patients with advanced liver metastases (clinical risk score [CRS] of 3–5), were treated with highly effective chemotherapy, proving respectability and survival rate were better than expected. Neoadjuvant chemotherapy has helped achieving control of the CRLM in more than 80% of cases, and of the primary tumour (as well as of invaded lymph-nodes) in more than 60% of cases [12]. A total of 92 patients have been now managed by a reversed treatment, and seven patients demonstrated complete histological responses of all metastases after chemotherapy.

The possibility that pCR of rectal cancer may occur without neoadjuvant radiation therapy is an intriguing hypothesis, which could promote the use of neoadjuvant chemotherapy alone also for non-metastatic colorectal cancer. The described patient with rectal cancer and liver metastasis was included in a “reversed” management protocol, aiming at treating the disease by chemotherapy first, and further resecting the liver metastases and the primary rectal cancer sequentially [9-11]. This unique type of management allowed for the assessment of the pathological response to chemotherapy alone.

## Case presentation

A 66-year old man presented with an adenocarcinoma of the rectum located 10 cm from the anal verge (uT3N1) (Figure 1). Thoraco-abdominal PET/CT scan revealed nine liver metastases (Figure 2). There were two lesions in the segment III, three in segment IV, one between segment V and VII, and three in segment VI. The carcinoembryonic antigen (CEA) was 8.3 μG/L. The clinical risk score was of two according to Fong’s classification (positive lymph node status, and multiple synchronous liver metastases).

**Figure 1:** **Radiological findings of the primary tumour.** CT scan and Pet-scan of the rectal tumour prior to chemotherapy.

**Figure 2:** **Computed tomography scan of liver metastases prior and after surgery: axial view A– H).** Liver metastases in all liver segments except segment 1. **I)** CT scan after surgery. extended right hepatectomy showing no recurrence.

Neoadjuvant chemotherapy consisted in a combination of oxaliplatin, 5-fluorouracil, irinotecan, leucovorin and bevacizumab (OCFL-B). Our strategy aimed at controlling the metastatic disease and performing liver surgery prior to rectal surgery, according to a “reversed” protocol previously described [9,11]. After three cycles, the patient did not report rectal bleeding anymore, and a major response of the liver metastases was documented on magnetic resonance imaging (MRI); all nine secondary tumours had decreased in size. After a right portal vein embolization, an extended right liver lobectomy with the local resection of two lesions in segment III was performed. On the final histopathological analysis, all lesions were fibrotic nodules, devoid of any viable cancer cells and compatible with previous metastases.

One month after liver surgery, a rectoscopic examination showed a near-total response of the primary rectal adenocarcinoma, which convinced the colorectal surgeon to proceed with pelvic surgery without preoperative radiation therapy. A low anterior resection of the rectum was carried out. Macroscopically, a fibrous scar was observed at the level of the previously documented tumour, and the histological examination of the surgical specimen did not reveal any malignant cells in the rectal wall as well as in the mesorectum. All 15 removed lymph nodes were free of tumour, and the final tumour stage was therefore ypT0N0M0 (Figure 3).

**Figure 3:** **Radiological appearance, operative specimen and histological profile of the primary tumour. A**. Pre-treatment PET scan showing hypermetabolic lesion of the mid rectum. **B**. Operative specimen of low anterior resection showing a fibrous scar in the mid rectum. **C**. Histological analysis of the operative specimen, showing the absence of tumour cells and the presence of fibrous tissue within the partially reepithelialised rectal wall.

This response was associated to an excellent clinical outcome: although the patient initially presented with bilobar liver metastases, he is currently alive without signs of recurrence five years after surgery. This confirms the advantages of preoperative chemotherapy and resection of colorectal liver metastasis to achieve pathologic response and hence predicts the survival rates [13].

## Conclusion

The current standard of care of patients with locally advanced rectal cancer includes the use of neoadjuvant chemoradiotherapy. Overall, 10–20% of patients achieve a complete rectal pathological response after chemoradiation. Some investigators have even demonstrated a sustained clinical response in the absence of rectal resection, with a low recurrence rate of 4.6%, and five-year overall and disease-free survival rates of 96 and 72% [14,15].

Despite these benefits, pelvic radiotherapy is linked to a number of limitations. It induces a peri-rectal inflammation, and the use of chemotherapy-only could make surgery easier, with higher chances of achieving a resection with appropriate margins by a minimally invasive approach. The use of radiotherapy in the management of rectal cancer is making another curative pelvic radiation impossible for potential prostatic, gynecological, bladder or anal cancer. In addition, it has long-term impact on anorectal, urinary and sexual function [16,17]. Finally, the recent improvements in the management of rectal cancer, including chemoradiotherapy and total mesorectal excision, have no impact on known or microscopic distant metastases.

The present patient with pCR received a chemotherapy combining oxaliplatin, 5-fluorouracil, irinotecan, leucovorin and bevacizumab. Oxaliplatin-based neoadjuvant chemotherapy, currently mainly used in stage IV patients, may represent an attractive alternative to the neoadjuvant radiation therapy for rectal cancer. Induction chemotherapy has the added advantage of earlier administration of systemic therapy and may improve the control or the prevention of distant metastasis.

Prospective randomized studies should be carried out to demonstrate effectiveness of systemic therapy into combined-modality programs and to evaluate the benefit of chemotherapy alone in selected patients with stages II-III rectal adenocarcinoma with or without distant metastasis.

## Consent

“Written informed consent was obtained from the patient for publication of this Case report and any accompanying images. A copy of the written consent is available for review by the Editor of this journal.”

## Abbreviations

CRC: Colorectal cancer; CRLM: Colorectal liver metastasis; 5-FU irinotecan: Oxaliplatin; OCFL-B: Leucovorin and bevacizumab; TME: Total mesorectal excision; CRT: Chemoradiotherapy; pCR: Pathologic complete response; CEA: Carcinoembryonic antigen; MRI: Magnetic resonance imaging.

## Competing interests

The authors declare that they have no competing interests.

## Authors’ contributions

LRB, AR, GM, PM, PG performed the clinical follow-up of the patient. GM, PG performed the surgery. CT, TT, PG and SN have made substantial contributions to conception and design, or acquisition of data, or analysis and interpretation of data. Furthermore, all authors have been involved in revising the manuscript critically for important intellectual content read and approved the final manuscript.

## Pre-publication history

The pre-publication history for this paper can be accessed here:

http://www.biomedcentral.com/1471-2482/14/4/prepub

## References

[B1] FerlayJShinHRBrayFFormanDMathersCParkinDMGLOBOCAN 2008 v2.0, Cancer Incidence and Mortality Worldwide: IARC CancerBase No. 10 [Internet]2010Lyon, France: International Agency for Research on CancerAvailable from: http://globocan.iarc.fr

[B2] BrayFRenJSMasuyerEFerlayJEstimates of global cancer prevalence for 27 sites in the adult population in 2008Int J Cancer2013132511331145doi: 10.1002/ijc.27711. Epub 2012 Jul 2610.1002/ijc.2771122752881

[B3] BeartRWJrMultidisciplinary management of patients with advanced rectal cancerClin Cancer Res20071322 Pt 26890s6893s1800679510.1158/1078-0432.CCR-07-1135

[B4] CervantesARodríguez-BraunENavarroSHernándezACamposSGarcía-GraneroEIntegrative decisions in rectal cancerAnn Oncol200718Suppl 912713110.1093/annonc/mdm30717631565

[B5] Rubbia-BrandtLGiostraEBrezaultCRothADAndresAAudardVSartorettiPDoussetBMajnoPESoubraneOChaussadeSMenthaGTerrisBImportance of histological tumor response assessment in predicting the outcome in patients with colorectal liver metastases treated with neo-adjuvant chemotherapy followed by liver surgeryAnn Oncol2007182993041706048410.1093/annonc/mdl386

[B6] AdamRWichertsDAde HaasRJAloiaTLeviFPauleBGuettierCComplete pathologic response after preoperative chemotherapy; myth or reality?J Clin Oncol2008261635164110.1200/JCO.2007.13.747118375892

[B7] O’NeillBDPBrownGHealdRJCunninghamDTaitDMNon-operative treatment after neoadjuvant chemoradiotherapy for rectal cancerLancet Oncol2007862563310.1016/S1470-2045(07)70202-417613424

[B8] Van CutsemEDicatoMHaustermansKArberNBossetJFCunninghamDThe diagnosis and management of rectal cancer: expert discussion and recommendations derived from the 9th world congress on gastrointestinal cancer, BarcelonaAnn Oncol2008 Jun19Suppl 618doi: 10.1093/annonc/mdn358. 200710.1093/annonc/mdn35818539618

[B9] MenthaGRothADTerrazSGiostraEGervazPAndresAMorelPRubbia-BrandtL‘Liver first’ approach in the treatment of colorectal cancer with synchronous liver metastasesDig Surg20082543043510.1159/00018473419212115

[B10] MenthaGTerrazSAndresATosoCRubbia-BrandtLMajnoPOperative management of colorectal liver metastasesSemin Liver Dis2013333262272doi: 10.1055/s-0033-1351785. Epub 2013 Aug 1310.1055/s-0033-135178523943106

[B11] MenthaGMajnoPEAndresARubbia-BrandtLMorelPRothADNeoadjuvant chemotherapy and resection of advanced synchronous liver metastases before treatment of the colorectal primaryBr J Surg20069387287810.1002/bjs.534616671066

[B12] GervazPRubbia-BrandtLAndresANeoadjuvant chemotherapy in patients with stage IV colorectal cancer: a comparison of histological response in liver metastases, primary tumors, and regional lymph nodesAnn Surg Oncol201017102714271910.1245/s10434-010-1056-620405223

[B13] DG 3rdBKishiYMaruDMKopetzSChunYSOvermanMJFogelmanDEngCChangDZWangHZorziDRiberoDEllisLMGloverKYWolffRACurleySAAbdallaEKVautheyJNPathologic response to preoperative chemotherapy: a new outcome end point after resection of hepatic colorectal metastasesClin Oncol2008263353445351doi: 10.1200/JCO.2008.17.5299. Epub 2008 Oct 2010.1200/JCO.2008.17.529918936472

[B14] Habr-GamaAPerezROS˜ao Juli˜aoGPProscurshimIGama-RodriguesJNonoperative approaches to rectal cancer: a critical evaluationSemin Radiat Oncol20112123424910.1016/j.semradonc.2011.02.01021645869

[B15] Glynne-JonesRHughesRCritical appraisal of the ‘wait and see’ approach in rectal cancer for clinical complete ressponders after chemoradiationBr J Surg2012997897909doi: 10.1002/bjs.8732. Epub 2012 Apr 2710.1002/bjs.873222539154

[B16] GervazPAWexnerSDPembertonJHPelvic radiation and anorectal function: introducing the concept of sphincter-preserving radiation therapyJ Am Coll Surg200219538739410.1016/S1072-7515(02)01308-X12229948

[B17] BujkoKNowackiMPNasierowska-GuttmejerAMichalskiWBebenekMKryjMLong-term results of a randomized trial comparing preoperative short-course radiotherapy with preoperative conventionally fractionated chemoradiation for rectal cancerBr J Surg2006931215122310.1002/bjs.550616983741

